The article "Clinical application of expectorant therapy in chronic inflammatory airway diseases (Review)" was published in 2014. Journal: Exp Ther Med.

# Clinical application of expectorant therapy in chronic inflammatory airway diseases (Review)

**DOI:** 10.3892/etm.2014.1494

**Published:** 2014-01-21

**Authors:** TING ZHANG, XIANGDONG ZHOU

**Affiliations:** Department of Respiratory Medicine, The Second Affiliated Hospital, Chongqing Medical University, Chongqing 400010, P.R. China

**Keywords:** airway mucus hypersecretion, chronic inflammatory airway disease, expectorant therapy

## Abstract

Airway mucus hypersecretion is a significant clinical and pathological feature of chronic inflammatory airway diseases. Its clinical presentations include recurrent coughing and phlegm. Airway mucus is closely associated with the occurrence, development and prognosis of chronic inflammatory airway diseases and critically affects the lung function, quality of life, hospitalization rate and mortality of patients with chronic inflammatory airway diseases. Therefore, expectorant therapies targeting the potential mechanisms of mucus hypersecretion have been the focus of numerous studies. Conventional expectorants are mainly mucoactive medicines, including nausea-stimulating expectorants, mucolytics, mucokinetics, and proteases and nucleases. In addition, certain traditional Chinese herbal medicines and non-mucoactive agents, including muscarinic acetylcholine receptor antagonists, corticosteroids, leukotriene receptor antagonists and macrolide antibiotics, have also shown expectorant effects. Several novel medicines for expectorant therapy have emerged, including cholesterol-lowering statins, epidermal growth factor receptor tyrosine kinase inhibitors, phosphodiesterase-4 inhibitors, stanozolol, surfactants, flavonoids, tachykinin receptor antagonists, protease inhibitors, cytokine antagonists and purinergic agonists. With the increasing number of multidisciplinary studies, the effectiveness of expectorant therapy for the treatment of chronic inflammatory airway diseases has been confirmed. Therefore, the development of novel expectorants and the standardization of expectorant therapy are the direction and focus of future studies, thus benefiting patients who have a chronic inflammatory airway disease.

## Introduction

Airway mucus hypersecretion is one of the important clinical and pathological features of chronic inflammatory airway diseases, including chronic obstructive pulmonary disease (COPD), bronchial asthma, bronchiectasis and cystic fibrosis (1–3). Long-term and repeated inflammatory stimuli of chronic airway inflammation induce the metaplasia of goblet cells, as well as the hyperplasia and hypertrophy of submucosal glands, causing a ‘secretory hyperresponsiveness’ that leads to impaired mucociliary clearance. Consequently, excessive mucus is more difficult to expel and is retained in the airways to form mucous plugs, which worsen the obstruction of the already narrowed airway and increase the colonization by pathogenic bacteria. These events may lead to persistent inflammation, sustained hypoxia, deterioration of the condition of a patient or even mortality (4–6). It has become increasingly clear that airway mucus hypersecretion is not only a clinical symptom but also an independent risk factor for disease progression and the poor prognosis of patients with chronic inflammatory airway diseases (7–9). Therefore, chronic inflammatory airway diseases with airway mucus hypersecretion has become a central issue in a number of studies (10–13). In the present study, the significance of expectorant therapy and the classification of common and novel expectorants are briefly reviewed.

The article "Clinical application of expectorant therapy in chronic inflammatory airway diseases (Review)" was published in 2014. Journal: Exp Ther Med.

## 2. Pathological changes of airway mucus hypersecretion and the association with respiratory diseases

Airway mucus is a heterogeneous mixture of glycoproteins, non-glycoprotein-like proteins, lipids, minerals, water and other compounds. Although the components and corresponding proportions in airway mucus vary greatly under different conditions, mucin, a highly glycosylated macromolecule, is always the major component and determines the hydrophilic and viscoelastic properties of airway mucus. The apparently elevated glycosylation and sulfation of mucus during chronic airway inflammation significantly increases the viscosity and acidity of airway mucus, making it immobile in the airway and thus more difficult to expel, which further aggravates the airway obstruction (14–16). A long-term study conducted by the European Community Respiratory Health Survey II revealed that in individuals with secretory hyperresponsiveness symptoms, including chronic cough and phlegm, the incidence of COPD is 2.88-fold higher than that in the general population and is not associated with smoking exposure (17). Burgel and Martin also confirmed that the incidence of acute exacerbation and readmission was markedly increased in patients with COPD with a cough and expectoration (9). Vestbo and Hogg identified that anti-inflammatory treatment alone was insufficient for the treatment of chronic inflammatory airway diseases, whereas expectorant therapy was not only able to significantly alleviate the clinical symptoms but also helped to reduce the respiratory inflammatory response (18). Delmotte *et al* determined that inflammatory cytokines, such as tumor necrosis factor-α, significantly enhanced the enzymatic activity of sulfotransferases and glycosyltransferases, which is consistent with the observation of increased glycosylation of mucin in patients with an inflammatory airway disease (19). A follow-up study, based on 101 patients with COPD (GOLD stage III–IV) who underwent lung volume reduction surgery, revealed that the severity of the airflow limitation induced by mucus hypersecretion was closely associated with the mortality of patients (20). Therefore, airway mucus hypersecretion plays an important role in the occurrence and development of chronic inflammatory airway diseases, and has been identified to be associated with the lung function, quality of life, hospitalization rate and mortality of patients with chronic inflammatory airway diseases. Consequently, expectorant therapy that is based on the potential mechanism of mucus hypersecretion has become an important target for the treatment of chronic inflammatory airway diseases.

The article "Clinical application of expectorant therapy in chronic inflammatory airway diseases (Review)" was published in 2014. Journal: Exp Ther Med.

## 3. Classification and mechanisms of common expectorants

Clinically available expectorant medicines are aimed at inhibiting the production and secretion of mucins, reducing the viscoelasticity of mucus, rehabilitating the normal structure and function of the mucus layer, improving mucociliary clearance and accelerating the transport of mucus. Accordingly, they are known as mucoactive agents (21,22), and are further divided into: i) Nausea-stimulating expectorants, such as guaifenesin; ii) mucolytics, such as ambroxol, which cleave mucopolysaccharide fibers, and N-acetylcysteine (NAC) and carbocisteine, which cleave disulfide bonds; iii) mucokinetics, such as myrtle oil, a powerful thinner of hardened mucus; and iv) proteases and nucleases, such as α-chymotrypsin. Of these classes, mucolytics and mucokinetics are primarily used, particularly ambroxol which accounts for almost 70% of the expectorant treatment in China (23).

As the most extensively used expectorant medicine in clinical practice in China, ambroxol has a very wide range of effects on the respiratory system. It is able to reduce the viscosity of sputum by inducing the bronchial glands to secrete serum and breaking up the mucopolysaccharide fibers of the mucin, which facilitates the penetration of antibiotics into the mucus and improves the local antibacterial effect. Simultaneously, ambroxol also induces alveolar type II cells to synthesize and secrete pulmonary surfactants that reduce the adhesion of the mucus to the cilia and accelerate the transport of mucus in the airway, which helps to expel the sputum and increase the airway mucosal clearance. In addition, ambroxol has specific antitussive, antioxidant and anti-inflammatory effects, along with a relatively significant inhibitory effect on histamine-induced constriction of the bronchial smooth muscle. Furthermore, it may also be used to prevent hyaline membrane disease in premature infants and to alleviate nitrosourea-induced pulmonary toxicity during the chemotherapy of malignant brain tumors (24,25).

The article "Clinical application of expectorant therapy in chronic inflammatory airway diseases (Review)" was published in 2014. Journal: Exp Ther Med.

As a mucolytic agent, the clinical efficacy of NAC has gained recognition and attention. It reduces the viscosity of mucus by cleaving the disulfide bonds of mucins and the DNA fibers in the purulent sputum, leading to its efficacy under conditions where general expectorant medicines are ineffective. It also accelerates the ciliary movement within airway mucosa and stimulates the gastro-pulmonary vagal reflex, thereby promoting the excretion of mucus. In addition, NAC has comprehensive antioxidant, anti-inflammatory, anti-injury, anti-lipid oxidation, anti-platelet aggregation, anti-mutagenesis and vasodilatory activities, and is able to protect anti-protease activity and inhibit allergic reactions, among others. (26–28). Pela *et al* demonstrated that the prolonged treatment of patients with COPD with NAC (400 mg/day for six months) led to a significant improvement in the forced expiratory volume in 1 sec and maximum expiratory flow at 50% of the forced vital capacity, accompanied by a significant reduction in exacerbations of 41% (29). Similarly, Gerrits *et al* concluded that a daily intake of 400 mg NAC has a significant protective effect and reduces the readmission rate of patients with COPD by 30% (30). In addition to being a safe and efficacious expectorant medicine, NAC has been extensively used to treat pulmonary diseases including emphysema, tuberculosis, fibrous alveolitis and primary pulmonary amyloidosis, as well as diseases of the cardiovascular and central nervous system and acquired immune deficiency syndrome (31).

Carbocisteine, as a mucoregulatory agent, recovers the viscoelasticity of normal mucus and enhances mucociliary clearance via interactions between the disulfide bonds of mucin and the carboxymethyl structure of the agent. The antioxidant and anti-inflammatory protective effects of carbocisteine on bronchial cells are also relevant to its efficacy in the treatment of chronic airway inflammatory diseases (32). The PEACE study on the efficacy of carbocisteine has shown that, although carbocisteine did not significantly improve the lung function and blood oxygen saturation of patients with COPD, the medicine significantly reduced the frequency of acute exacerbations of COPD (AECOPD) and improved health-related quality-of-life scores compared with those of the control group. Therefore, the authors recommended that carbocisteine is used for the prevention and treatment of AECOPD (33). Other studies have also indicated that carbocisteine is able to improve the quality of life of patients with COPD (34,35).

The article "Clinical application of expectorant therapy in chronic inflammatory airway diseases (Review)" was published in 2014. Journal: Exp Ther Med.

Although the longstanding and popular therapeutic option for the treatment of chronic inflammatory airway diseases is mucoactive medicines, numerous non-expectorant agents have also received great attention as a type of mucus therapy. The agents that are commonly available for clinical use include muscarinic receptor blockers, glucocorticosteroids, leukotriene receptor antagonists, macrolide antibiotics, 2–3% hypertonic sodium chloride and 2–7% hypertonic sodium bicarbonate solution. Each of them inhibits the excessive production and/or secretion of airway mucins via different mechanisms despite their common treatment functions (22,36).

## 4. Chinese herbal expectorants

The role of herbal medicine is significant in expectorant management. Balloon flower, rhizoma arisaematis, Caladium, Polygala and Aster are commonly adopted for expectorant therapy. Triterpenoid saponins are considered as the major effective ingredients. These Chinese herbal medicines are mainly nausea-stimulating expectorants, which induce mild nausea by stimulating the gastric mucosa and stimulate the respiratory gland cells to increase the secretion of thinner sputum, thus facilitating its expulsion. Chinese herbal expectorants have a confirmed therapeutic effect, and their clinical application is promising. However, a number of issues remain to be improved, such as variations to prescriptions and over-dispersive studies. Therefore, further exploration of highly efficacious and rapid-onset agents is required for the development of novel medications for oral administration (37–39).

## 5. Novel types of expectorants

### Statin-like cholesterol-lowering medicines

Statins, such as simvastatin, are a class of medicines used to lower cholesterol levels. A number of studies have identified that they are also able to modulate airway inflammatory processes by inhibiting the expression of a variety of inflammatory factors and inducing the apoptosis of inflammatory cells, which helps to inhibit inflammation-induced airway mucus hypersecretion. Further, the anti-inflammatory effect of statins has been verified to be independent of their lipid-lowering role. A few studies have suggested that the anti-inflammatory effect of statins is directly associated with their function of promoting the apoptosis and clearance of inflammatory cells (40–42). It has also been demonstrated that statins are able to reduce the morbidity and mortality of patients with COPD (43,44), suggesting that the combined effects of statins on COPD may lead to them becoming a novel therapy option for chronic airway inflammatory diseases.

The article "Clinical application of expectorant therapy in chronic inflammatory airway diseases (Review)" was published in 2014. Journal: Exp Ther Med.

### Epidermal growth factor receptor (EGFR) tyrosine kinase inhibitors

The EGRF signaling pathway is a common pathway for numerous inflammatory mediators leading to mucus overproduction in human airways. Therefore, blocking this pathway provides a novel treatment target for airway mucus hypersecretion and reduces sputum retention. Clinical case studies have identified that the selective EGFR tyrosine kinase inhibitor gefitinib (Iressa), which is used to treat non-small-cell lung cancer, markedly inhibited airway mucus hypersecretion in patients with lung cancer. Further, the suppressive effect on airway mucus hypersecretion occurred prior to and more markedly than the inhibition of the growth of the tumor (45–47).

### Phosphodiesterase-4 inhibitors

As a major metabolic enzyme of cyclic adenosine monophosphate during the inflammatory response, phosphodiesterase-4 plays an important regulatory role in the synthesis and release of airway non-adrenergic non-cholinergic neurotransmitters. Suppression of phosphodiesterase-4 reduces the release of inflammatory mediators and downregulates inflammatory responses and thereby the airway mucus hypersecretion. The novel selective phosphodiesterase-4 inhibitors cilomilast and roflumilast inhibit the activation of numerous inflammatory and immune cells in chronic inflammatory diseases. Therefore, their anti-inflammatory effect indicates positive prospects for phosphodiesterase-4 inhibitors in the management of airway mucus hypersecretion (48–50)

### Stanozolol-related medicines

Stanozolol-related medicines, including erdosteine, fudosteine and lifusteine, play important roles in regulating the composition, properties and motion of mucus. These medicines are able to promote mucociliary transport, reduce the stimulation of mucus secretion, protect α1-antitrypsin protease against the activation of protease, specifically human neutrophil elastase, and significantly increase the concentration of antimicrobial agents in the sputum (as well as synergistically regulating the local activity of those agents). They are have anti-inflammatory activity, aid mucosal repair, suppress goblet cell hyperplasia and promote serous secretion (51–54). Therefore, this class of medicines is ideal for the comprehensive treatment of chronic inflammatory airway diseases, particularly COPD.

### Surfactants

Tyloxapol is representative of this class of medicines and decreases the surface tension of sputum, thereby reducing its viscosity and facilitating expectoration.

### Flavonoids

Flavonoids are natural ingredients that are extracted from plants with similar biological activities. A considerable number of studies conducted on animals, as well as *in vitro,* have demonstrated the diverse beneficial biological activities of flavonoids, including anti-inflammatory, antioxidative and antibacterial activities and the induction of apoptosis. All of these effects are beneficial for the prevention and treatment of pulmonary diseases. Theaflavins, exocarpium citri grandis, Forsythia, breviscapine, naringenin, farrerol and quercetin are typical clinically used flavonoids and flavonoid-containing therapeutic agents (55–57). Due to their low costs and high availability from natural sources, these medicines have great potential for development as medicines for chronic inflammatory airway diseases.

The article "Clinical application of expectorant therapy in chronic inflammatory airway diseases (Review)" was published in 2014. Journal: Exp Ther Med.

### Tachykinin receptor antagonists

Tachykinins, including neuropeptide A, neuropeptide B and substance P, are a class of non-adrenergic non-cholinergic neurotransmitter that can mediate neurogenic mucin secretion via neurokinin 1 receptors. A long-acting tachykinin receptor antagonist, MEN11467, inhibits the secretory response (58), suggesting its therapeutic potential for airway mucus hypersecretion

### Protease inhibitors

Neutrophil elastase is the most powerful inflammatory stimulus currently known to cause the significant synthesis and secretion of mucin (59). Studies on airway mucus hypersecretion in asthma have revealed that the neutrophil elastase inhibitors ONO-5046 and ICI 200,355 are able to suppress ozone-induced and ovalbumin sensitization-induced goblet cell hypersecretion and neutrophil accumulation, respectively (60,61). The protease inhibitor sivelestat is now available for the clinical treatment of acute pulmonary injury. Furthermore, the future treatment of airway diseases with sivelistat (or Sivelestat), a small molecule inhibitor of neutrophilelastase, is planned (62).

### Cytokine antagonists

Various types of cells and cytokines are involved in the complex pathological process of chronic airway inflammation and stimulate the abnormal production and secretion of mucin in bronchial epithelial cells. Bacillus Calmette-Guérin (BCG), as a nonspecific immunomodulator, is a type of powerful immune stimuli. It increases the expression levels of Th1-like cytokines (e.g. interferon-γ and interleukin (IL)-12), inhibits the expression of Th2-like cytokines, reduces the accumulation and infiltration of eosinophils in airways, and suppresses the hyperplasia and metaplasia of goblet cells as well as the resultant mucus production and secretion. Therefore, BCG achieves preventive and therapeutic results (63). Furthermore, studies on antagonists of other types of cytokines (e.g. IL-4, IL-9 and transforming growth factor-β) are in progress (64–66).

### Purinergic agonists

The purine-sensitive receptor, P2Y2, has a comprehensive role in the regulation of the steady state of the airway mucus layer. The P2Y2 receptor, when activated, enhances the transmembrane movement of water molecules, thins out mucins and accelerates cilial transport mobility. P2Y2 receptor agonists include purine nucleoside triphosphates, pyrimidine nucleosides and INS365 (67). Studies have indicated that inhaled pyrimidine nucleosides and INS365 are capable of accelerating the mucus flow rate in airways and enhancing mucociliary clearance; another P2Y2 agonist, INS37217, has activity similar to that of pyrimidine nucleosides (68,69).

The article "Clinical application of expectorant therapy in chronic inflammatory airway diseases (Review)" was published in 2014. Journal: Exp Ther Med.

## 6. Summary

With the continued exploration of the role of airway mucus hypersecretion in the pathogenesis of chronic inflammatory airway diseases, the results confirm from an evidence-based medicine point of view that patients with chronic inflammatory airway diseases benefit from treatment with expectorants (70). The crucial role of timely and effective expectorant intervention for the treatment of chronic airway inflammatory disease has been widely accepted by clinicians. However, controversies remain over the applicable subjects, the reasonable dosage and the duration of treatment, among other therapeutic considerations. The phenomenon of chronic airway mucus hypersecretion (presenting as a cough and expectoration) is ubiquitous in all chronic airway inflammatory diseases. Therefore, a study has suggested that therapies targeting mucus hypersecretion in chronic airway inflammation should be recommended regardless of the presence of a chronic cough and expectoration (9). Thus, future studies on the mechanism of expectorant medicines and the exact role expectorant medicines should play in the standard treatment of chronic airway inflammatory diseases are required. The development of novel expectorant medicines and an optimal therapeutic regimen is required.
